The article "Hypertension and diabetes mellitus are associated with high FIB-4 index in a health checkup examination cohort without known liver disease" was published in 2022. Journal: BMC Gastroenterol.

# Hypertension and diabetes mellitus are associated with high FIB-4 index in a health checkup examination cohort without known liver disease

**DOI:** 10.1186/s12876-022-02575-5

**Published:** 2022-11-21

**Authors:** Shunsuke Sato, Hidehiko Kawai, Sho Sato, Hirohiko Iwasaki, Masashi Omori, Yuji Kita, Yuji Ikeda, Takahito Awatsu, Ayato Murata, Gentaro Taniguchi, Yuji Shimada, Takuya Genda

**Affiliations:** 1 Department of Gastroenterology and Hepatology, Juntendo University Shizuoka Hospital, 1129 Nagaoka, Izunokuni, Shizuoka 410-2295 Japan; 2 Fuji Town Medical Center, 12-12 Fujicho, Shizuoka, Fuji 416-0915 Japan

**Keywords:** Diabetes mellitus, Fibrosis-4 index, health check-up examination, Hypertension, Liver fibrosis, Non-alcoholic fatty liver disease

## Abstract

**Background:**

Non-alcoholic fatty liver disease (NAFLD) is usually asymptomatic and lacks a specific biomarker; therefore, many individuals might remain undiagnosed even with advanced liver fibrosis. The aim of this study was to clarify the prevalence and clinical features of subjects with a high risk of advanced liver fibrosis in the general population, using the Fibrosis-4 (FIB-4) index.

**Methods:**

We retrospectively investigated 6,087 subjects without known liver disease who had participated in an annual health checkup examination. We analyzed the factors associated with high FIB-4 index (≥ 2.67) using a logistic regression analysis.

**Results:**

Among the 6,087 subjects, 76 (1.2%) had high FIB-4 index. Multivariate analysis identified hypertension (odds ratio [OR]; 9.040; 95% confidence interval [CI], 4.081–20.024; *P* < 0.001) and diabetes mellitus (OR = 4.251; 95% CI, 1.773–10.193; *P* = 0.001) as important risk factors for high FIB-4 index. The rates of hypertension and diabetes mellitus in subjects with high FIB-4 index were 78.9% and 23.7%, respectively. No significant association was observed between obesity or large waist circumference and high FIB-4 index. A history of cardiovascular disease was significantly more common in subjects with high FIB-4 index. These results were also observed in subjects with normal liver function test.

**Conclusions:**

The present study revealed that approximately 1% of the general Japanese population has a high risk of advanced liver fibrosis. Many of these patients had hypertension and/or diabetes mellitus. Our findings suggest that there are many undiagnosed patients NAFLD with risk of advanced liver fibrosis in the general population.

## Background

Non-alcoholic fatty liver disease (NAFLD) is rapidly becoming the main cause of liver cirrhosis and hepatocellular carcinoma (HCC), owing to recent changes in lifestyle and dietary habits [1, 2]. The global prevalence of NAFLD has reached 25.2% in the general population, and it is a growing public health problem worldwide [3]. In Japan, the prevalence of NAFLD is estimated to increase from 17.9% in 2016 to 18.8% in 2030; the incidence of decompensated cirrhosis is estimated to increase by 67%, and the incidence of HCC is estimated to increase by 44% from 2016 to 2030 [4]. However, many patients are presumed to remain undiagnosed, even those with advanced liver fibrosis, since NAFLD is usually asymptomatic and shows only relatively normal or only mildly elevated liver enzyme levels.

The article "Hypertension and diabetes mellitus are associated with high FIB-4 index in a health checkup examination cohort without known liver disease" was published in 2022. Journal: BMC Gastroenterol.

In NAFLD, advanced liver fibrosis is well-known to be the most important prognostic factor for overall mortality [5, 6]. Recent international guidelines recommend that patients with NAFLD should be assessed for the presence of advanced liver fibrosis [7, 8]. Liver biopsy remains the gold standard for assessment of liver fibrosis, but it carries the risk of severe complications such as hemorrhage, high cost, and sampling variability [9]. Therefore, the Fibrosis-4 (FIB-4) index, one of the most common non-invasive fibrosis tests based on aspartate aminotransferase (AST), alanine aminotransferase (ALT), age and platelet counts, is often used for assessment liver fibrosis instead of lever biopsy. FIB-4 index was originally proposed to assess liver fibrosis in patients with human immunodeficiency virus and hepatitis C virus co-infection [10]. However, due to its low-cost, convenience and high negative predictive values, FIB-4 index was now recommended for use to rule out advanced liver fibrosis in general population, particularly for NAFLD and alcohol-related liver disease [11, 12].

In this study, we identified subjects with high FIB-4 index in a health checkup cohort without known liver disease, and clarified their prevalence and clinical features.

## Methods

### Subjects

We registered 16,248 subjects who participated in an annual health checkup examination at the Fuji Town Medical Center in Shizuoka from April 2019 to March 2020. Of these subjects, 10,065 were excluded owing to lack of blood examination (*n* = 2,217) or platelet count data (*n* = 7,848). Therefore, we included 6,183 for whom we were able to calculate the FIB-4 index. The excluded subjects had a median age of 46 years and 49.6% were male, showing no significant differences from the corresponding characteristics of the included subjects (*P* = 0.051 and *P* = 0.399, respectively). In addition, we excluded 27 subjects with hepatitis B or C virus infection or a history of other chronic liver diseases such as autoimmune hepatitis, primary biliary cirrhosis, hemochromatosis, and Wilson’s disease, and 69 subjects who consumed alcohol > 60 g/day. Finally, 6,087 subjects were retrospectively analyzed in the present study. The study protocol was approved by the Ethics Committee of Juntendo University Shizuoka Hospital (No. 829), and the study was performed in accordance with the 2013 revision of the Declaration of Helsinki.

The article "Hypertension and diabetes mellitus are associated with high FIB-4 index in a health checkup examination cohort without known liver disease" was published in 2022. Journal: BMC Gastroenterol.

### Data collection

We obtained information regarding age, sex, smoking habits, current alcohol consumption (daily alcohol drinking ≥ 30 g for male and ≥ 20 g for female), present illnesses, past history of cardiovascular disease (CVD), and treatment using a self-report questionnaire. In addition, basic anthropometric measurements such as height, weight, body mass index (BMI), waist circumference, systolic blood pressure, and diastolic blood pressure were obtained. The following laboratory data were also collected: AST, ALT, gamma-glutamyl transpeptidase (GGT), albumin, high-density lipoprotein (HDL) cholesterol, low-density lipoprotein (LDL) cholesterol, triglyceride, fasting plasma glucose, hemoglobin A1c (HbA1c), uric acid, white blood cell count, hemoglobin, and platelet count. Biochemical tests had been performed after 12 h of fasting.

### Assessment of the risk of advanced liver fibrosis

The FIB-4 index was calculated as previously described (age [years] × AST [IU/L] / (platelet count [10^9^/L]) × ALT (IU/L)^1/2^] [10]. The subjects were categorized into three groups, as previously described: <1.30 (low risk), 1.30-2.67 (intermediate risk), and >2.67 (high risk of advanced liver fibrosis).

### Definition of obesity, large waist circumference, and comorbidity status

Obesity was defined as a BMI ≥ 25.0 kg/m^2^ based on the World Health Organization Asia–Pacific guidelines [13]. A large waist circumference was defined as ≥ 85 cm in males and ≥ 90 cm in females based on the diagnostic standards of metabolic syndrome [13]. Habitual drinking was defined as consumption of ethanol/day > 20 g and > 30 g for female and male, respectively [14]. Diabetes mellitus was defined as a fasting plasma glucose level ≥ 126 mg/dL, HbA1c ≥ 6.5%, casual plasma glucose level ≥ 200 mg/dL, or present treatment using antihyperglycemic medicine [15]. Hypertension was defined as systolic blood pressure ≥ 140 mmHg and/or diastolic blood pressure ≥ 90 mmHg or present treatment for hypertension based on the Japanese Society of Hypertension guidelines [16]. Dyslipidemia was defined as triglycerides ≥ 150 mg/dL, HDL cholesterol < 40 mg/dL, LDL cholesterol ≥ 140 mg/dL, or present treatment for dyslipidemia based on the Japanese Atherosclerosis Society guidelines [17]. Hyperuricemia was defined as a serum uric acid level ≥ 7.0 mg/dL, or present treatment for hyperuricemia based on the Japanese Society of Gout and Nucleic Acid Metabolism [18]. CVD was defined as history of ischemic heart disease or stroke.

The article "Hypertension and diabetes mellitus are associated with high FIB-4 index in a health checkup examination cohort without known liver disease" was published in 2022. Journal: BMC Gastroenterol.

### Statistical analyses

Categorical data were compared using the chi-squared method. Continuous variables were analyzed using the Mann–Whitney U test. Factors associated with advanced liver fibrosis were determined using logistic regression analysis. Odds ratios and 95% confidence intervals (CI) were calculated. Statistical significance was set at *P* < 0.05. All statistical analyses were performed using the PASW Statistics 18 software (IBM SPSS, Chicago, IL, USA).

## Results

### Baseline characteristics

The baseline characteristics of the study participants are summarized in Table 1. Among the 6,087 subjects, the percentages of those aged < 30 years, those in their 30 s, 40 s, 50 s, and 60 s, and those aged ≥ 70 years were 12.3%, 18.6%, 26.9%, 22.9%, 12.9%, and 6.3%, respectively. The proportion of participants with obesity was 25.5%, and the proportion of those with a large waist circumference was 25.9%. A total of 4,524 subjects (74.3%) showed normal serum ALT levels (upper limits of 19 and 30 IU/L for female and male, respectively). The rates of hypertension, diabetes mellitus and dyslipidemia were 31.7%, 5.2%, and 45.2%, respectively.

**Table 1:** Baseline characteristics

Variables	
Age (year)	47 (11-89)
Sex (Male / Female)	3,076 / 3,011
Smoking (%)	21.0
Habitual drinking (%)	12.4
BMI (kg/m^2^)	22.4 (10.6-61.1)
Waist circumference (cm)	79.9 (58.0-152.5)
Systolic blood pressure (mmHg)	125 (77-244)
Diastolic blood pressure (mmHg)	74 (34-140)
Fasting plasma glucose (mg/dL)	92 (57-321)
HbA1c (%)	5.6 (4.4-14.6)
Triglyceride (mg/dL)	81 (16-1454)
LDL cholesterol (mg/dL)	122 (25-335)
HDL cholesterol (mg/dL)	63 (11-158)
Uric acid (mg/dL)	5.2 (0.4-11.6)
Albumin (g/dL)	4.4 (3.4-5.3)
AST (IU/L)	20 (5-233)
ALT (IU/L)	18 (3-561)
GGT (IU/L)	22 (5-1,086)
Platelet counts (× 10^4^/μL)	24.9 (2.9-59.5)
Hemoglobin (g/dL)	14.2 (7.0-19.7)
White blood cell (/μL)	5,400 (1,100-17,800)
FIB-4 index	0.84 (0.17-6.82)
Hypertension (%)	31.7
Diabetes mellitus (%)	5.2
Dyslipidemia (%)	45.2
Hyperuricemia (%)	8.2

Data are expressed as median (range), *ALT* Alanine aminotransferase, *AST* Aspartate aminotransferase, *BMI* Body mass index, *FIB-4* Fibrosis-4, *GGT* Gamma-glutamyl transpeptidase, *HbA1c* Hemoglobin A1c, *HDL* High-density lipoprotein, *LDL* Low-density lipoprotein

### Distribution of the FIB-4 index

The distribution of the FIB-4 index is shown in Fig. 1. The median FIB-4 index was 0.84. Among all subjects, 4,828 (79.3%), 1,183 (19.4%), and 76 (1.2%) showed FIB-4 index < 1.30, 1.30–2.67, and ≥ 2.67, respectively.

The article "Hypertension and diabetes mellitus are associated with high FIB-4 index in a health checkup examination cohort without known liver disease" was published in 2022. Journal: BMC Gastroenterol.

**Fig. 1:** Distribution of FIB-4 index in subjects who participated in an annual health checkup examination. Abbreviations: FIB-4, Fibrosis-4

### Comparison of baseline characteristics according to FIB-4 index

A comparison of the baseline characteristics according to the FIB-4 index is shown in Table 2. In the subjects with high FIB-4 index (≥ 2.67), age, AST, ALT, GGT, creatinine level, the prevalence of habitual drinking, and the complication rate of hypertension or diabetes mellitus, were significantly higher than in those with FIB-4 index < 2.67. In contrast, the smoking rate, albumin level, platelet count, and white blood cell count, were significantly lower than in those with FIB-4 index < 2.67. There were no significant differences in BMI, waist circumference, the prevalence of obesity or large waist circumference, and dyslipidemia such as triglyceride or LDL cholesterol, between the two groups. The prevalence of subjects with elevated serum ALT levels with FIB-4 index ≤ 1.30, 1.30–2.67, and ≥ 2.67 was 25.8%, 24.3%, and 38.2%, respectively (Fig. 2).

**Table 2:** Comparison of baseline characteristics according to FIB-4 index

Variables	FIB-4 < 2.67 (Low-intermediate risk of advanced liver fibrosis) *N* = 6011	FIB-4 ≥ 2.67 (High risk of advanced liver fibrosis) *N* = 76	*P* value
**Age** (year)	47 (11-89)	72 (41-88)	< 0.001^†^
**Male** (%)	50.4	57.9	0.120^‡^
**Smoking** (%)	21.2	7.9	0.002^‡^
**Habitual drinking** (%)	12.7	25.7	0.002^‡^
**BMI** (kg/m^2^)	22.4 (10.6-61.1)	22.4 (16.8-31.2)	0.948^†^
**Obesity** (%)	25.7	26.3	0.493^‡^
**Waist circumference** (cm)	80.0 (54.1-152.5)	79.8 (57.5-112.5)	0.229^†^
**Large waist circumference** (%)	26.3	34.2	0.080^‡^
**Systolic blood pressure** (mmHg)	124 (77-244)	138 (105-174)	< 0.001^†^
**Diastolic blood pressure** (mmHg)	74 (34-140)	78 (51-106)	0.019^†^
**Fasting plasma glucose** (mg/dL)	92 (57-295)	104 (79-321)	< 0.001^†^
**HbA1c** (%)	5.6 (4.4-14.6)	5.7 (5.1-8.6)	0.001^†^
**Triglyceride** (mg/dL)	80 (16-1,454)	87 (30-432)	0.280^†^
**HDL cholesterol** (mg/dL)	63 (11-158)	38 (38-103)	0.364^†^
**LDL cholesterol** (mg/dL)	122 (25-335)	121 (61-178)	0.148^†^
**Uric acid** (mg/dL)	5.2 (0.4-11.6)	5.2 (2.5-8.4)	0.627^†^
**Albumin** (g/dL)	4.4 (3.4-5.3)	4.3 (3.7-4.9)	0.040^†^
**AST** (IU/L)	20 (5-203)	28 (16-233)	< 0.001^†^
**ALT** (IU/L)	18 (3-561)	20 (7-212)	0.009^†^
**GGT** (mg/dL)	22 (5-1,086)	27 (10-313)	< 0.001^†^
**Platelet counts** (× 10^4^/μL)	25.0 (8.5-59.5)	14.8 (2.9-28.6)	< 0.001^†^
**Hemoglobin** (g/dL)	14.2 (7.0-19.7)	14.0 (8.1-17.0)	0.152^†^
**White blood cell** (/μL)	5,400 (1,900-17,800)	4,500 (1,100-13,900)	< 0.001^†^
**Creatinine** (mg/dL)	0.76 (0.30-14.1)	0.79 (0.50-1.30)	0.010^†^
**Hypertension** (%)	31.3	78.9	< 0.001^‡^
**Diabetes mellitus** (%)	5.0	23.7	< 0.001^‡^
**Dyslipidemia** (%)	45.1	52.6	0.115^‡^
**Hyperuricemia** (%)	11.5	9.1	0.352^‡^

Data are expressed as median (range), †Mann-Whitney U-test, ‡Chi-squared test. *ALT* Alanine aminotransferase, *AST* Aspartate aminotransferase, *BMI* Body mass index, *Fib-4* Fibrosis-4, *GGT* Gamma-glutamyl transpeptidase, *HbA1c* Hemoglobin A1c, *HDL* High-density lipoprotein, *LDL* Low-density lipoprotein

The article "Hypertension and diabetes mellitus are associated with high FIB-4 index in a health checkup examination cohort without known liver disease" was published in 2022. Journal: BMC Gastroenterol.

**Fig. 2:** Prevalence of subjects with normal serum ALT levels according to FIB-4 index. Abbreviations: FIB-4, Fibrosis-4; ALT, alanine aminotransferase

### Risk factors associated with high FIB-4 index

To identify the risk factors associated with high FIB-4 index, logistic regression analysis was performed (Table 3). Univariate analysis revealed that the absence of smoking habits, habitual drinking, hypertension or diabetes mellitus, lower albumin levels, white blood cells, and higher GGT levels, were associated with high FIB-4 index. Multivariate analysis identified four independent risk factors: hypertension (odds ratio [OR] = 9.040; 95% confidence interval [CI], 4.081–20.024; *P* < 0.001), diabetes mellitus (OR = 4.251; 95% CI, 1.773–10.193; *P* = 0.001), albumin levels (OR = 0.265; 95% CI, 0.083–0.841; *P* = 0.024) and white blood cell count (OR = 0.999; 95% CI, 0.999–1.000; *P* < 0.001).

**Table 3:** Factors associated with high FIB-4 index

Variables	Univariate analysis		Multivariate analysis	
	**OR (95%CI)**	**P value**	**OR (95%CI)**	***P* value**
**Sex (Male vs. Female)**	0.740 (0.468-1.170)	0.198		
**Smoking**	0.318 (0.138-0.734)	0.007		
**Habitual drinking**	2.338 (1.381-3.956)	0.002		
**Obesity**	1.034 (0.619-1.728)	0.899		
**Large waist circumference**	1.456 (0.903-2.347)	0.123		
**Hypertension**	8.217 (4.721-14.302)	< 0.001	9.040 (4.081-20.024)	< 0.001
**Diabetes mellitus**	5.935 (3.454-10.200)	< 0.001	4.251 (1.773-10.193)	0.001
**Dyslipidemia**	1.354 (0.861-2.131)	0.190		
**Albumin**	0.268 (0.087-0.828)	0.022	0.265 (0.083-0.841)	0.024
**GGT**	1.006 (1.003-1.008)	< 0.001		
**White blood cell**	0.999 (0.999-1.000)	< 0.001	0.999 (0.999-1.000)	< 0.001
**Hemoglobin**	0.919 (0.799-1.058)	0.240		
**Creatinine**	1.218 (0.903-1.643)	0.197		

*BMI* Body mass index, *FIB-4* Fibrosis-4, *GGT* Gamma-glutamyl transpeptidase

### Prevalence of metabolic factors according to FIB-4 index

The associations of metabolic factors such as obesity, large waist circumference, hypertension, diabetes mellitus, and dyslipidemia, with the FIB-4 index are shown in Fig. 3. Among them, the rates of hypertension and diabetes mellitus increased with FIB-4 index. The complication rates of hypertension were 26.1%, 52.4%, and 78.9% in subjects with FIB-4 index ≤ 1.30, 1.30–2.67, and ≥ 2.67, respectively (*P* < 0.001). The complication rates of diabetes mellitus were 3.8%, 9.8%, and 23.7% in subjects with FIB-4 index ≤ 1.30, 1.30–2.67, and ≥ 2.67, respectively (*P* < 0.001). In addition, the number of subjects with both hypertension and diabetes mellitus was significantly higher among those with high FIB-4 index (Fig. 4). These correlations were also observed in subjects with normal serum ALT levels (Fig. 5).

The article "Hypertension and diabetes mellitus are associated with high FIB-4 index in a health checkup examination cohort without known liver disease" was published in 2022. Journal: BMC Gastroenterol.

**Fig. 3:** Complication rate of metabolic factors according to FIB-4 index. **a** Obesity; **b** Large waist circumference; **c** Hypertension; **d** Diabetes mellitus; and **e** Dyslipidemia. Abbreviations: FIB-4, Fibrosis-4

**Fig. 4:** Complication rate of hypertension and diabetes mellitus according to FIB-4 index. Abbreviations: FIB-4, Fibrosis-4

**Fig. 5:** Complication rate of metabolic factors according to FIB-4 index in subjects with normal serum ALT levels. **a** Obesity; **b** Large waist circumference; **c** Hypertension; **d** Diabetes mellitus; and **e** Dyslipidemia. Abbreviations: FIB-4, Fibrosis-4; ALT, alanine aminotransferase

### History of cardiovascular disease according to FIB-4 index

Since hypertension and diabetes mellitus are important risk factors for cardiovascular events, we investigated the association between the FIB-4 index and a history of cardiovascular disease. Among the subjects with FIB-4 index ≤ 1.30, 1.30–2.67, and ≥ 2.67, 1.6%, 5.4%, and 9.3% had a history of cardiovascular disease, respectively (*P* < 0.001, Fig. 6). These results were also observed in subjects with normal serum ALT levels (Fig. 7).

**Fig. 6:** Complication rate of cardiovascular disease according to FIB-4 index. Abbreviations: FIB-4, Fibrosis-4

**Fig. 7:** Complication rate of cardiovascular disease according to FIB-4 index in subjects with normal serum ALT levels. Abbreviations: FIB-4, Fibrosis-4; ALT, alanine aminotransferase

## Discussion

Advanced liver fibrosis is the most important prognosis factor across etiologies [12]. The present study revealed that approximately 20% of the general Japanese population has an intermediate risk of advanced liver fibrosis, and approximately 1% has a high risk of advanced liver fibrosis. These results were confirmed by a recent systematic review that showed that the prevalence of liver fibrosis varied between 0.7% and 25.7%, the prevalence of advanced liver fibrosis varied between 0.9% and 2.0%, and cirrhosis varied between 0.1% and 1.7% [19].

The present study was revealed that many subjects had high risk of advanced liver fibrosis complicated by diabetes mellitus and hypertension. Metabolic factors such as diabetes mellitus and hypertension, are considered the most important comorbidities of NAFLD. Diabetes mellitus is the most important risk factors of NAFLD and clinical predictor of adverse outcomes such as developing clinical decompensation and hepatocellular carcinoma [20, 21]. In addition, patients with hypertension show a higher prevalence of NAFLD and advanced liver fibrosis, and NAFLD increases the risk of incident hypertension [22, 23]. Many subjects at high risk of advanced liver fibrosis had hypertension and diabetes mellitus, suggesting that there are many patients who have NAFLD, but have not yet been diagnosed. More importantly, a significant association between high FIB-4 levels and hypertension or diabetes mellitus was found in subjects with normal ALT levels. These results suggest the existence of NAFLD in patients with advanced liver fibrosis, even in those with apparently normal liver function test. In addition, subjects with high FIB-4 index showed low white blood cell counts and albumin levels, which might have been related to splenomegaly and portal hypertension due to advanced liver fibrosis.

The article "Hypertension and diabetes mellitus are associated with high FIB-4 index in a health checkup examination cohort without known liver disease" was published in 2022. Journal: BMC Gastroenterol.

Furthermore, our study showed that a history of cardiovascular disease was significantly higher in subjects with high FIB-4 index. A recent meta-analysis showed that patients with NAFLD had a higher risk of fatal cardiovascular events than those without NAFLD, and that the progression of liver fibrosis was an independent risk factor for the development of cardiovascular events [24].

In addition to hypertension and diabetes mellitus, both obesity and a large waist circumference are fundamental components of metabolic syndrome and are closely associated with NAFLD. However, our study showed no association between obesity or large waist circumference and high FIB-4 index. Although the reason for this discrepancy remains unclear, it may be associated with non-obese or lean NAFLD. In fact, it was estimated that approximately 19.2% of NAFLD patients are lean, and 40.8% are non-obese [25]. Recently, a patatin-like phospholipase domain-containing protein 3 (PNPLA3) gene polymorphism has been shown to be associated with NAFLD and to play an important role in NAFLD development in the non-obese population [26]. Interestingly, the PNPLA3 rs738409 GG genotype is more prevalent in Asians than in Caucasians [27]. This might explain the absence of association between obesity or a large waist circumference and advanced liver fibrosis observed in our study.

Finally, this study has several limitations that need to be acknowledged. First, we could not use liver biopsies to perform histological evaluation. In the future, liver stiffness measurements using transient elastography, and more accurate testing for liver fibrosis will be required. Second, we could not evaluate fatty liver using B-mode ultrasound imaging. Third, this study was a single-center study in Japan; therefore, it remains unclear whether these findings are applicable to other countries.

The article "Hypertension and diabetes mellitus are associated with high FIB-4 index in a health checkup examination cohort without known liver disease" was published in 2022. Journal: BMC Gastroenterol.

## Conclusions

In summary, our study suggests that many potential patients have not yet been diagnosed with NAFLD. Early identification of individuals at high risk of advanced liver fibrosis is clinically important. Primary care physicians play an important role in the diagnosis and management of NAFLD; however, it remains uncertain how to implement screening, and which patients in the general population should be referred to a hepatologist. Our findings suggest that to identify individuals at high risk of advanced liver fibrosis, we should target those with lifestyle-related diseases, particularly hypertension and diabetes mellitus.

## Data Availability

All data generated or analyzed during this study are included in this published article.

## Abbreviations

ALT: Alanine aminotransferase
AST: Aspartate aminotransferase
CI: Confidence interval
FIB-4: Fibrosis-4
GGT: Gamma-glutamyl transpeptidase
HCC: Hepatocellular carcinoma
HDL: High-density lipoprotein
LDL: Low-density lipoprotein
NAFLD: Non-alcoholic fatty liver disease.
PNPLA3: Patatin-like phospholipase domain-containing protein 3
